The article "Ethical Conflict and Knowledge Hiding in Teams: Moderating Role of Workplace Friendship in Education Sector" was retracted in 2025. Reasons: unreliable results or conclusions; a conflict of interest; concerns about the peer review; concerns about the citations.

# Ethical Conflict and Knowledge Hiding in Teams: Moderating Role of Workplace Friendship in Education Sector

**DOI:** 10.3389/fpsyg.2022.824485

**Published:** 2022-02-10

**Authors:** Shuo Xing

**Affiliations:** Department of Marxism, Hunan University of Science and Technology, Xiangtan, China

**Keywords:** ethical conflicts, knowledge hiding, ethical value congruence, shared ethical priority, teams

## Abstract

Ethical conflicts arise when there is no unity between the team members and shared ethical priorities. This study aimed to identify the relationship between ethical value unity, team knowledge hiding, the relationship between the lack of shared ethical priorities and the team knowledge hiding. Workplace friendship was taken as a moderating variable to check its regulating role between the ethical conflicts and the team knowledge hiding. Data of this study were collected from the staff working in different colleges and universities. There are a total of 480 responses collected through convenience sampling technique and analyzed under a five-point Likert scale. The partial least squares-structural equation modeling (PLS-SEM) technique is used in this study. The key reason was that this approach has the fewest requirements for data normality and is a better tool for evaluating exploratory connections empirically. The output of the measurement model assessment confirms that all measurement scales are reliable. The result indicates that there was a significant and positive relationship between ethical value congruence and knowledge hiding. It was also established that there was a relationship between lack of shared ethical priorities and knowledge hiding. Workplace friendship moderated the relationship between ethical conflicts and team knowledge hiding. This study extends the literature on ethical conflict and knowledge hiding behavior. This study highlights that one of the main reasons for knowledge hiding behavior at the team level in the organization is which helps the business practicians for a design of an effective strategy to mitigate the knowledge hiding behavior in the organization.

## Introduction

Individuals are confronted with ethical conflicts challenges when their values, ethics, and morality clashes with the experience. In certain condition, there are very difficult to discriminant between right and wrong and have to choose between two evils. Conflicts of this nature might occur on an individual, professional, or social level. When it comes to ethical conflicts, whether the aims justify the methods is frequently raised. For instance, doing what is ethically correct might have a negative impact, while doing what is morally wrong or immoral can benefit. Individuals, communities, and nations must decide which option is more ethical in light of these factors. Furthermore, the moral perspective may or may not be supported by facts. For example, Parents may refuse to give their kids a life-saving blood transfusion because they feel it is unethical. Traditional, textbook examples of hypothetical moral dilemmas can be used to investigate the ethical conflict. The lifeboat example is one such scenario in which one person must be thrown overboard for the rest to live.

The article "Ethical Conflict and Knowledge Hiding in Teams: Moderating Role of Workplace Friendship in Education Sector" was retracted in 2025. Reasons: unreliable results or conclusions; a conflict of interest; concerns about the peer review; concerns about the citations.

The role model test asks if it would bother a person if her role model were aware of her behaviors or decisions. The golden rule test asks if a person is fine with her decision influencing others, in the same manner, it affects her (Brown et al., 2021). Apart from the current advancement in company management, ethical conflicts have grown in power and taken on new shapes and forms. The most popular and heated topics are corporate interest, ethics, and transparency (Pennington et al., 2021). The organization’s ethical atmosphere cannot be described as excellent. Many ethical difficulties may be noticed in many enterprises and management, such as illegal practices, cybercrime, lack of workplace safety, such as legal responsibility and other fraudulent practices. Following social media’s creation and widespread adoption, concerns about cyber ethics have grown significantly (Nuseir and Ghandour, 2019). Consequently, ethical difficulties in modern management are becoming a major issue. Ethical dilemmas and their practices in various organizations have recently drawn attention since they are now easily disclosed on social media (Brown et al., 2021). It may have a detrimental impact on the workplace, with organizations losing their reputation and popularity, resulting in a decline in client numbers, lost business, and revenue decreases (Avotra et al., 2021a). Various examples of firms failing and closing due to ethical difficulties, such as a major American energy company (Brown et al., 2021). Workplace ethical conflict has previously been studied in arguments over work duties, processes, and personal relationships (Kim et al., 2015). On the other hand, conflicts frequently entail issues of right and wrong; yet, ethical conflict is noticeably lacking from the literature. Brown et al. (2020) proposed the concept of ethical conflict, developed and validated a measure of it, and investigated its specific implications on workplace outcomes using moral convictions theory.

Ethical conflict is a two-edged sword, it is linked to poor team dynamics, such as lower group satisfaction, viability, cohesiveness, psychological safety; increased negative emotions; and perceived goal difficulties (Brown et al., 2021). Ethics is the central axis that helps organizations, corporations, and enterprises to achieve favorable financial outcomes, job balance, and well-being by balancing risk. On the other hand, a lack of ethical principles application might have a detrimental impact on individuals, resulting in harm, severe penalties, and even bankruptcy. There have been several examples involving a lack of ethics that reputable experts have highlighted throughout the years. Furthermore, in one of his studies, researchers examine the vast differences in business conduct, demonstrating significant ethical case responses (Fichter, 2018; Sison et al., 2019). Ethics is a subject that has persisted throughout history, manifesting itself in many sorts of organizations and civilizations. Ethics has consequences, either when it is applied for the common good, resulting in harmony, trust, solidarity, and peace, or when it is not applied, resulting in suffering and destruction to human beings. Ethics is a wide concept that occurs in many aspects of life, including business and administration, and is crucial in all areas, including leadership, teamwork, and successful communication (Tammany et al., 2019).

The article "Ethical Conflict and Knowledge Hiding in Teams: Moderating Role of Workplace Friendship in Education Sector" was retracted in 2025. Reasons: unreliable results or conclusions; a conflict of interest; concerns about the peer review; concerns about the citations.

In general, value congruence leads to increased and improved communication and fewer misunderstandings and conflicts. As a result, when followers disagree with their leaders about what is essential and ethically suitable, they are less inclined to seek and accept their opinion on ethical matters actively. In contrast, followers who feel their leaders share comparable ethical ideals and underlying ideas about ethically good and wrong are more inclined to see and accept them as valid ethical role models worthy of following (Cheng et al., 2019). Ethical conflict arises with an employee’s personal beliefs collide with the organization’s, negative consequences such as stress, lack of organizational commitment, absenteeism, and turnover can ensue. Individuals should work together to achieve the objective. A team is developed when individuals possessing multiple talent and skills work together to attain the same goals. Team members are jointly responsible for doing everything it takes to attain the goal. Team sizes vary, but due to the inefficiency of a big group of individuals working together in practice, people typically refer to groups of less than 20 people when they talk about teams (Brown et al., 2021).

However, strictly speaking, there are no restrictions on the size of a team. Even a major firm with hundreds of employees might claim to operate as a team or with a sense of camaraderie (Ogunyemi, 2019). Prioritization should be unbiased and regard persons as equals as per ethical views. According to a growing agreement, the goals should be to promote health maximization, equitable distribution, and poverty prevention. Three ethical priority-setting criteria emerge from these guiding principles: cost-effectiveness, priority to the poor, and financial risk protection. Prioritizing services based on the cost-effectiveness of novel interventions vs. current standards is critical, given that extending and enhancing people’s lives have both direct and indirect benefits. Furthermore, this is not always the case, the most cost-effective programmers frequently benefit the poorest and give the most financial risk protection. Cost-effectiveness, however, cannot be the only consideration. Prioritizing the poor is crucial since it will benefit them more than the well-off and will lessen unjust inequities. Those with the most severe and biggest individual illness burdens and those who are poor or otherwise disadvantaged are considered the worst-off. Because the most cost-effective treatments do not necessarily help the poorest people, services aimed at them should be given more on priority (Ogunyemi, 2019). Human beings, according to Maslow, have an inbuilt need to fulfill wants ranging from the most basic to the most complicated, such as friendships. Workplace friendship, also known as an informal interpersonal relationship at work, is a close and voluntary bond between coworkers that differs from the formal one, such as leader-subordinate or instrumental. Workplace friendship has both a socio-emotional and a utilitarian purpose in fostering a productive and friendly work environment. Some empirical studies show that workplace friendship affects turnover intention, emotional commitment, information sharing, and job performance, whereas qualitative studies look at both positive and negative effects.

The article "Ethical Conflict and Knowledge Hiding in Teams: Moderating Role of Workplace Friendship in Education Sector" was retracted in 2025. Reasons: unreliable results or conclusions; a conflict of interest; concerns about the peer review; concerns about the citations.

Despite all of this past study, there is still no conclusive empirical evidence for determining when and how workplace friendship would result in a positive outcome, such as information sharing among team members (Eva et al., 2019). Employee knowledge concealment, defined as the deliberate withholding of information when it is sought, happens often and is a serious problem in the workplace. Unfortunately, many corporate structures and practices, such as employee competitiveness, encourage information concealing among employees. Because previous information hiding research has demonstrated that this issue has negative consequences for employees, such as lower individual creativity and strained relationships, additional study into the characteristics that might help avoid knowledge hiding is needed. Information hiding can help us understand many social interactions in organizations if we know it at the dyadic level; however, knowledge hiding does not always happen sequentially at the dyadic level. Rather, many debates and exchanges occur in groups, and there may be information concealed at the group level. As a result, we develop the term team knowledge hiding to explain what happens when a team has a high level of knowledge concealing. Examining hidden knowledge at the group level might reveal new information about employee actions and dynamics at work (An et al., 2021; Xiaolong et al., 2021; Yingfei et al., 2021). So ethical conflict, its constituents, such as ethical value congruence, ethical priorities and their relationship with the detrimental effects of knowledge hiding among the teams, and the moderating role of workplace friendship have a lot to evaluate in this study. So our study revolved around certain objectives to estimate the impact of ethical conflicts on team knowledge hiding discussed above.

## Review of Literature

### Social Exchange Theory

Social exchange theory, Blau (1964) is the principal lenses through which the theoretical framework of this study was to be examined. The central theme is that individual behaviors maximize positive experiences and minimize negative experiences. Similarly, Dalton (1972) identifies three types of reciprocity: generalized, balanced, and negative. Generalized reciprocity refers to a positive exchange relationship between employer and employee, whereas negative reciprocity refers to a negative exchange between two parties governed by mistrust and self-interest (Liden et al., 1997). Balanced reciprocity refers to a neutral economic exchange relationship (Dalton, 1972). They are drawing on social exchange theory (Blau, 1964). Humans, according to the first premise, want to seek out rewards and avoid penalties. One main motivation of the individual to perform certain action to maximize profit in the minimum expenses. Another principle is that a person enters a transaction with the goal of maximizing profit at the lowest possible expense as the individual is motivated by what is in it for me?. A third assumption is that people analyses the profit and expense of doing something before doing it. This theory determines that people realize that the payoff will differ from one person to the next and over time (Cook and Rice, 2006). The main principles of social exchange theory form a fundamental foundation, namely, that one size does not fit all. These degrees of anticipation are frequently used in combination with another basic idea of the theory’s functionality: the cost–benefit analysis. This is likely the most well-known aspect of the theory since it offers a “give and take” measure that can be used to assess how much effort one side is putting into the relationship. This theory element’s costs are items that a person would consider a negative in a relationship.

The article "Ethical Conflict and Knowledge Hiding in Teams: Moderating Role of Workplace Friendship in Education Sector" was retracted in 2025. Reasons: unreliable results or conclusions; a conflict of interest; concerns about the peer review; concerns about the citations.

An acquaintance who borrows money often or a spouse who regularly fails to perform his household responsibilities might rack up a significant bill. Benefits, under this perspective, are characteristics that an individual may consider to be favorable. Applying the metrics that construct social exchange theory together may be a fantastic tool for analyzing connections and human behavior from a sociological approach (Cook and Rice, 2006). Sociologists can use the dynamics that make this theory function to construct their own ideas and conceptions about how humans interact regarding knowledge sharing or hiding due to ethical conflicts (Ali et al., 2021).

### Affective Events Theory

According to the Effective events theory, emotional states impact job performance, leading to knowledge sharing in team and pleasure. The hypothesis describes the link between employees internal factors, such as temperament, feelings, conflicts, intellect, and responses to workplace situations. Theorists suggest that employee mood and emotion explain productive work behaviors, but cognitive-based actions are good indicators of job happiness. Simply put, how people manage problems at work is influenced by their emotions and mood (Avotra et al., 2021a). The following elements form the foundation of the theory, that is, features of the working environment, working events, personal dispositions or conflicts and response to the events of the work (Cropanzano et al., 2016). The links between components connected with work, such as job characteristics, job expectations, and needs for emotional labor, and their influence on employment results, are known as aspects of the working environment. Job happiness is influenced by one’s autonomy and flexibility in determining one’s own work schedule. Personal dispositions or conflicts describe the connection between a worker’s temperament and attitude and the impact it has on workplace events and how they affect quality of work life. The five-factor personality dimension that includes conscientiousness, agreeableness, openness to experience, neuroticism, and extraversion, demonstrates individual characteristics and their influence on work performance and pleasure. While negative occurrences are recorded less frequently than happy events, they have a greater influence on mood. These might be both beneficial and bad in nature. In forecasting intentions toward poor-performing workers, emotions have a higher effect than attributions or expectancies (Cropanzano et al., 2016). Our research which is about ethical conflicts, such as ethical value congruence and the lack of shared ethical priorities and their relationship with the negative attributes in a team, that is, knowledge hiding along with moderating role of workplace friendships, is supported by these two theories.

The article "Ethical Conflict and Knowledge Hiding in Teams: Moderating Role of Workplace Friendship in Education Sector" was retracted in 2025. Reasons: unreliable results or conclusions; a conflict of interest; concerns about the peer review; concerns about the citations.

### Relationship Between Ethical Value Congruence and Team Knowledge Hiding

Ethics experts recognize that relational processes are rooted in a social environment and will comprehend ethical principles in teams which requires examining both persons and their surroundings concurrently. Maintaining the constructive tension between individuals and their settings is especially urgent in ethical ideals (Albert et al., 2015). Individuals’ motivation hinders when they perceive the ethical difference between themselves and other team members to actively share information, resulting in poor information exchange evaluations within the team. According to one method, out-group individuals are perceived as less reliable sources of information, and ethically different people are deemed out-group members (van Knippenberg and Mell, 2016). Resultantly, messages from team members are more likely to be attended to and elaborated, and therefore more likely to affect the individual’s ideas and actions, than communications from non-team members.

According to a recent study, people are less likely to exchange knowledge with persons they believe different from themselves. The degree of similarity in ethical ideals among team members influences the willingness to share information (Crane et al., 2019). If a team has a value congruence issue, team members will likely be less receptive to other ideas and communicate less, interfering with productive group operations. Resultantly, in the negative association between diversity and performance, diversity research emphasizes the mediating function of ethical conflict of value congruence and team knowledge concealment, that is, team information utilization. Numerous studies have discovered that most forms of differences, particularly when they arise from deep-level traits like ethics, can lead to conflict, leading to knowledge hiding in the teams (Crane et al., 2019). This is a crucial component of the ethical values approach’s congruence component, which implies that these disparities lead to conflict and a lack of information sharing or knowledge concealment in teams, affecting team effectiveness (de Wit et al., 2012).

To put it another way, the notion or connection emphasizes the direct connection between ethical inconsistency, relational conflict, and knowledge concealment. Relationship conflict, which arises from personal inconsistency and unpleasant emotions, is particularly linked to poor team performance and group processes. Ethical disagreement among team members encourages adversarial or critical attributions for the actions of other team members (Kearney et al., 2009). Because they sense a danger or humiliation, team members are inclined to stop providing information or hide their knowledge in such situations. They are more likely to sense a threat of opportunism, which might discourage them from freely providing their data (Chowdhury, 2005). Taken together, we propose that the absence of ethical value congruence, as a result of ethical conflict, leads to the feeling that information is hidden more in the team. So, we proposed the following.

The article "Ethical Conflict and Knowledge Hiding in Teams: Moderating Role of Workplace Friendship in Education Sector" was retracted in 2025. Reasons: unreliable results or conclusions; a conflict of interest; concerns about the peer review; concerns about the citations.

*H_1_*: *There is a relationship between ethical value congruence and team knowledge hiding*

### Relationship Between Shared Ethical Priorities and Team Knowledge Hiding

A team is developed when individuals with the necessary skills and expertise work to attain a certain common objective. The individual should work together to achieve certain common objectives. Team members are jointly responsible for doing everything it takes to attain the goal. Team sizes vary, but due to the inefficiency of a big group of individuals working together in practice, people typically refer to groups of less than 20 people when they talk about teams. However, strictly speaking, there are no restrictions on the size of a team. Even a major firm with hundreds of employees might claim to operate as a team or with a sense of togetherness. Occasionally, team members have a say in who they work with, while other times they are “forced” to work together. In any scenario, forming a team needs trust and honesty. To put it another way, if individuals are to work successfully together, ethics are required (Ogunyemi, 2019). Knowledge hiding practices can range from modest to significant, such as disregarding a simple request to concealing essential or strategic knowledge (Khalid et al., 2018).

There are certain causes of reasoned knowledge hiding like protecting secrets or concealing private information; employees rarely participate in rationalized knowledge hiding in response to an ethical conflict between shared ethical values defined by leaders (Serenko and Bontis, 2016). Knowledge concealing is frequently a passive reaction to a circumstance, such as harsh supervision; it is not always meant to do direct harm to other members of the organization (Mitchell and Ambrose, 2007). We suggest that social exchange theory can explain the link between a lack of shared ethical objectives and information concealment practices. There is not much research available on the direct relations between ethical conflict of lack of shared ethical priority between teams and the team knowledge hiding but there is a great scope for finding the relation between them. So, we hypothesized the following to test the significance of this kind of relationship.

The article "Ethical Conflict and Knowledge Hiding in Teams: Moderating Role of Workplace Friendship in Education Sector" was retracted in 2025. Reasons: unreliable results or conclusions; a conflict of interest; concerns about the peer review; concerns about the citations.

*H_2_*: *There is a relationship between shared ethical priority and team knowledge hiding*

### Moderating Role of Workplace Friendship

Generally, workplace friendships in team knowledge hiding studies have not been a topic of debate in the past but as a team, friendships among the members sharing the common workplace could be the regulating one between ethical conflicts and the knowledge hiding at team level. As, workplace friendship could be beneficial or detrimental by the side in the transfer of knowledge which leads to the failure or success of the teamwork. Sometimes, sharing friendships at the workplace boosts the efficiency of the work and sometimes reduces the work’s efficiency, so it was much necessary to define the regulating role of workplace friendship among the ethical conflicts and the team knowledge hiding. Extra shifts spent on the job, demanding work programmers, and an understanding of how vital working with a group is for the organization’s activities and advantages and supporting it all contribute to organizations taking friendship interactions into account. Within the workplace, many levels of friendship can be created. In the workplace, friendships exist between subordinates and superiors, vice versa, and between coworkers.

Interpersonal interactions have been categorized as work relationships and friendships in research of the workplace social context. A work relationship is a job connection that involves an organizational-role view, comes from work-related concern, and is mandated by job design or thought required for job accomplishment, work-role needs, or work objectives. Employees, on the other hand, form friendships of their own choice. Without any external limits or pressures, the partners may interact freely with one another. Friendship is seen as a human tie that requires a personalistic perspective and interactions based on a personal concern to meet the personal requirements of both the self and the partners. Individual obligations to one another take precedence over meeting work/organizational demands in friendship. As a result, the impact of friendship on workers will differ from that of a work connection, and there is an area dedicated to friendship concerns in the organizational study on relationships (Methot et al., 2016).

The article "Ethical Conflict and Knowledge Hiding in Teams: Moderating Role of Workplace Friendship in Education Sector" was retracted in 2025. Reasons: unreliable results or conclusions; a conflict of interest; concerns about the peer review; concerns about the citations.

These factors can have various effects on an individual’s career, performance, motivation, and organizational atmosphere and performance. By describing workplace friendship as non-private, voluntary workplace connections, it was stated that it manifested itself as mutual trust, fancy, commitment, common interests, and values. Employees’ ties and friendships with their coworkers were said to provide an emotional support system and take conventional supervisory and mentoring roles. Indeed, these studies emphasized the importance of analyzing the antecedents that facilitated the creation of workplace friendships and intimate ties for various reasons, including internal employee rewards, lowering and balancing work-related stress, and so on (Yavuzkurt, 2020). In research conducted by Yavuzkurt (2020), more than 250 secondary school teachers participated in the study, which attempted to uncover the link between workplace friendship views and job happiness.

The descriptive and inferential statistical approaches were utilized in this investigation, which was planned using the relational screening model. Secondary school teachers were found to have a high level of internal job satisfaction and friendship opportunities. It was also shown that there were moderately favorable connections between teacher’s job happiness and their views of workplace friendships. It was discovered that teachers views of friendship opportunities impacted their job happiness substantially and beneficially.

As a moderator of intimate personal ties in the organization, workplace friendship may give psychological and behavioral support, such as trustworthiness and information sharing, that is beneficial to work. To put it another way, socializing with coworkers friends may be emotionally rewarding and increase employees psychological resources. Because of the peaceful, helpful, and pleasant atmosphere in which the individual is immersed, workplace friendship can drive employees to demonstrate interpersonal citizenship (Methot et al., 2016). It has been discovered that workplace friendship boosts a worker’s interpersonal energy, which leads to higher interpersonal engagement, using time-lagged, multi-source data across more than 600 individuals from several workgroups. Furthermore, they revealed the relationship between self-construal as a key moderating factor that influences a relationship’s saliency. Workplace friendship does have a larger favorable impact on someone’s interpersonal energy and hence interpersonal citizenship for employees with a relational-interdependent self-construal. Based upon the literature stating various roles of workplace friendships, we hypothesized the regulating or the moderating role of workplace friendships toward our goal of finding reasons of team knowledge hiding as follows.

The article "Ethical Conflict and Knowledge Hiding in Teams: Moderating Role of Workplace Friendship in Education Sector" was retracted in 2025. Reasons: unreliable results or conclusions; a conflict of interest; concerns about the peer review; concerns about the citations.

*H_3_*: *Workplace friendship moderate the relationship between ethical value congruence and team knowledge hiding*

*H_4_*: *Workplace friendship moderates the relationship between shared ethical priorities and team knowledge hiding*

A following conceptual model (Figure 1) has been formed based on the above literature and hypothesis.

**Figure 1:** Conceptual model.

## Methodology

### Population and Sampling

The population of this study is the staff working in colleges and universities of China. Team was made and segregated based on the nature of their work and specialization; then, data were collected based upon team level using a convenience sampling technique. Total 550 questionnaires were distributed among the staff, out of which 500 responses were received. However, 30 responses exclude due to missing values and outliers. So that the 480 responses are analyzed in this study. The response rate of this study is 90%. The total number of male respondents is 320 and female respondents are 180.

### Measures

Five-point Likert scale was used to measure all variables. Ethical value congruences were measured with a seven-item scale which was utilized (Thorne, 2010). A sample item includes “My firm share my value and companion for other.” Seven-item scale adapted from Thorne (2010) that was used for measuring lack of shared ethical priorities. Knowledge hiding was assessed with the 12-item scale that was used to measure knowledge hiding behavior construct by Connelly et al. (2012). Sample item include “In a specific episode in which a particular coworker requested knowledge from you and you declined” and 06 items scale was used to assess workplace friendship. A sample item includes “I have the opportunity to get to know my coworkers.” Firstly, the questionnaire was designed with the scale adapted from previous studies mentioned above as it has been checked and verified by linguistic and management specialists then the pilot study was conducted to measure the validity and reliability of construct before collecting data on a large level.

### Techniques

The (PLS-SEM) technique is used in this study. SmartPLS 3 version 2.7 was utilized to implement this approach. The key reason was that this approach has the fewest requirements for data normality and is a better tool for evaluating exploratory connections empirically. PLS-premier SEM’s sources have been followed in terms of data analysis and outcomes interpretation (Avotra et al., 2021b).

## Data Analysis and Results

Partial least squares-structural equation modeling analysis was used in this study for data analysis and to examine the theoretical framework. There are several reasons for using PLS-SEM analysis. This approach is best suited for testing the hypotheses and complex model. This technique is also suitable for identifying measurement errors and present correct estimation (Nawaz et al., 2019). This technique is effective for data analysis of simple and complex model and need no specific data normality conditions (Hao et al., 2020). PLS-SEM considers both measurement and structural models. SmartPLS software was used to perform data analysis which consists of two-stage. First measurement analysis was conducted to ensure the internal consistency and validity of data. Then, the structural model was examined to test the proposed hypotheses by using a bootstrapping technique.

The article "Ethical Conflict and Knowledge Hiding in Teams: Moderating Role of Workplace Friendship in Education Sector" was retracted in 2025. Reasons: unreliable results or conclusions; a conflict of interest; concerns about the peer review; concerns about the citations.

### Measurement Model

In the first step of the PLS-SEM construct, reliability, consistency, convergent, and discriminant validity were examined, known as measurement assessment model. First, factor loading of all the items of constructs was examined. Minimum acceptable factor loadings should be greater than 0.70 (Vinzi et al., 2010). However, some scholars suggest that even factor loadings greater than 0.50 are acceptable. According to Latif et al. (2020), instead of automatically removing factor loadings having low value, it was examined to check whether removing outer loadings helps increase the reliability, content validity, and convergent validity of the constructs. Therefore, factor loadings values range from 0.40 to 0.70 removed only if deletion of items helps to increase the value of composite reliability and average variance extracted (AVE). In this study, a few items of construct having less factor loading were deleted to be obtained to increase composite reliability and AVE (i.e., KH11, KH12, SEPR4, SEPR7, and EVC3).

Instrument reliability ensures that the indicators used to measure a construct are correct and valid. There are three methods to determine constructs internal consistency or reliability; Cronbach’s alpha and composite reliability. Table 1 illustrates the alpha value of all constructs greater than 0.700 and ranges from 0.789 to 0.939. Hence, internal consistency of construct was established. The second method to assess the internal consistency is Rho_A. Its value should be greater than 0.700 as recommended by Avotra et al. (2021a). The third method for assessing the internal reliability and consistency of a scale is composite reliability. Value of CR greater than the range between 0.60 and 0.70 is considered acceptable. It is highlighted that the composite reliability of each latent construct is above 0.70; thus, internal consistency is established. The AVE was examined to assess the convergent validity of the construct. The minimum threshold of AVE is equal to greater than 0.500 to determine the convergent validity of the construct.

The article "Ethical Conflict and Knowledge Hiding in Teams: Moderating Role of Workplace Friendship in Education Sector" was retracted in 2025. Reasons: unreliable results or conclusions; a conflict of interest; concerns about the peer review; concerns about the citations.

**Table 1:** Item loadings, reliability, and convergent validity.

Construct	Loadings	Alpha	Rho_A	CR	AVE
*Ethical value congruence*		0.852	0.860	0.900	0.694
EVC1	0.890				
EVC2	0.754				
EVC3	0.858				
EVC4	0.824				
EVC6	0.780				
*Lack of shared ethical priorities*		0.890	0.900	0.913	0.599
SEPR1	0.811				
SEPR2	0.777				
SEPR3	0.771				
SEPR4	0.758				
SEPR5	0.762				
SEPR6	0.768				
SEPR7	0.769				
*Knowledge hiding*		0.934	0.940	0.946	0.661
KH1	0.823				
KH2	0.865				
KH3	0.868				
KH4	0.847				
KH5	0.777				
KH6	0.855				
KH7	0.871				
KH8	0.802				
KH9	0.769				
KH10	0.767				
*Workplace friendship*		0.879	0.882	0.912	0.675
WP2	0.843				
WP3	0.789				
WP4	0.854				
WP5	0.825				
WP6	0.795				
WP6	0.671				

The coefficient of determination (*R*^2^) value of KH is 0.672 and predictive relevance (*Q*^2^) value is 0.513. AVE, average variance extracted; CR, composite reliability, EVC, ethical value congruences; KH, knowledge hiding; SEPR, lack of shared ethical priorities; WP, workplace friendship.

After establishing the reliability and convergence, the discriminant validity of the construct was examined. Discriminant validity refers to who two concepts are distinct to each other if two or more concepts are unique, then valid measures of each should not correlate high. There are three methods to investigate the discriminant validity of constructs, such as Fornell and Larcker, cross-loadings and Heterotrait-Monotrait (HTMT). The square root of AVE of each variable in the research model must be higher than the correlation of the same variable with others to determine the discriminant validity of the construct. Table 2 reflects that the square root of AVE of each construct is greater than the diagonal values below.

**Table 2:** Discriminant validity (Fornell and Larcker criterion).

	EVC	KH	SEPR	WP
EVC	0.833			
KH	0.625	0.813		
SEPR	0.418	0.663	0.774	
WP	0.405	0.611	0.587	0.822

EVC, ethical value congruences; KH, knowledge hiding; SEPR, lack of shared ethical priorities; WP, workplace friendship.

Another method to determine the discriminant validity of constructs is cross-loadings. Cross-loading helps assess if an item belonging to particular construct loads strongly onto its own parent construct instead of other constructs in the study. The results (Table 3) show that factor loadings of all the items is stronger on the underlying construct to which they belong instead of other constructs in the study (Wasko and Faraj, 2005).

The article "Ethical Conflict and Knowledge Hiding in Teams: Moderating Role of Workplace Friendship in Education Sector" was retracted in 2025. Reasons: unreliable results or conclusions; a conflict of interest; concerns about the peer review; concerns about the citations.

**Table 3:** Cross-loading.

	EVC	KH	SEPR	WP
EVC1	**0.890**	0.572	0.342	0.377
EVC2	**0.755**	0.459	0.291	0.244
EVC3	**0.858**	0.487	0.291	0.330
EVC4	**0.822**	0.551	0.455	0.383
KH1	0.504	**0.815**	0.534	0.515
KH2	0.484	**0.860**	0.607	0.598
KH3	0.539	**0.856**	0.553	0.492
KH4	0.512	**0.843**	0.525	0.480
KH5	0.444	**0.769**	0.515	0.438
KH6	0.523	**0.860**	0.575	0.512
KH7	0.553	**0.870**	0.575	0.552
KH8	0.569	**0.809**	0.560	0.501
KH9	0.434	**0.598**	0.374	0.347
SEPR1	0.316	0.462	**0.812**	0.457
SEPR2	0.319	0.469	**0.777**	0.478
SEPR3	0.288	0.450	**0.772**	0.371
SEPR4	0.251	0.433	**0.758**	0.370
SEPR5	0.274	0.400	**0.762**	0.386
SEPR6	0.373	0.648	**0.768**	0.526
SEPR7	0.389	0.618	**0.769**	0.523
WP2	0.347	0.543	0.518	**0.843**
WP3	0.284	0.449	0.453	**0.790**
WP4	0.344	0.484	0.468	**0.855**
WP5	0.374	0.534	0.478	**0.824**

Factor loadings of items with their construct are shown as bold and italic. EVC, ethical value congruences; KH, knowledge hiding; SEPR, lack of shared ethical priorities; WP, workplace friendship.

HTMT (Heterotrait-Monotrait Ratio) is the criteria to determine the discriminant validity. If the values of HTMT are higher which depicts the issues of discriminant validity in the constructs. The threshold value of HTMT is 0.9 which means two variables are correlated but not more than 0.90. Table 4 shows that all value of HTMT is less than 0.900 thus discriminant validity was established.

**Table 4:** HTMT (Heterotrait-Monotrait Ratio) of correlations.

	EVC	KH	SEPR	WP
EVC				
KH	0.699			
SEPR	0.463	0.700		
WP	0.462	0.669	0.646	

### Structural Model

In the second step, structural model was assessed by using structural equation modeling (SEM) technique as shown in Figure 2. In the structural model, *R*^2^, *Q*^2^, and the significance of paths were measured. Strength of each path measured by using *R*^2^ which is known as the goodness of model (Briones Peñalver et al., 2018). *R*^2^ of knowledge hiding is 0.627 as shown in Table 5 which means that all exogenous variables account for 62% variance in knowledge hiding. The structural model’s predictive relevance is estimated through the blindfolding technique with an omission distance of 7. The value of *Q*^2^ above 0 shows predictive accuracy (Hair et al., 2019). Table 5 shows that the *Q*^2^ value is above 0 which shows the predictive accuracy of the construct. The hypotheses testing was carried out using a bootstrapping technique, with a re-sample of the number of 5,000 bootstraps. H_1_ proposed that there is a relationship between ethical value congruence and knowledge hiding. The result indicates that there is a significant and positive relationship between ethical value congruence and knowledge hiding (*β* = 0.350, *t* = 11.606, *p* = 0.000). As a value of *p* < 0.05, therefore this hypothesis is accepted. H_2_ proposed that there is a relationship between Lack of shared ethical priorities and knowledge hiding. The result indicates that there is a relationship between lack of shared ethical priorities and knowledge hiding (*β* = 0.354, *t* = 10.734, *p* = 0.000). As a value of *p* < 0.05, therefore this hypothesis is accepted. H_3_ proposed that workplace friendship moderates the relationship between EVC and knowledge hiding. The result indicates that WPF significantly moderates the relationship between EVC and knowledge hiding (*β* = 0.050, *t* = 2.039, *p* = 0.045). As a value of *p* < 0.05, therefore this hypothesis is accepted. H_4_ proposed that workplace friendship moderates the relationship between Lack of shared ethical priorities and knowledge hiding. The result indicates that WPF significantly moderates the relationship between SEPR and knowledge hiding (*β* = 0.079, *t* = 2.659, *p* = 0.008). As a value of *p* < 0.05, therefore this hypothesis is accepted as shown in Table 6.

The article "Ethical Conflict and Knowledge Hiding in Teams: Moderating Role of Workplace Friendship in Education Sector" was retracted in 2025. Reasons: unreliable results or conclusions; a conflict of interest; concerns about the peer review; concerns about the citations.

**Figure 2:** Structural assessment model.

**Table 5:** Direct effects.

Hypotheses	Path	Beta coefficient	SD	*T* value	*p*	Decision
H1	EVC → KH	0.350	0.030	11.606	0.000	Supported
H2	SEPR → KH	0.354	0.033	10.734	0.000	Supported

**Table 6:** Moderation effects.

Hypotheses	Path	Beta coefficient	SD	*T* value	*p*	Decision
H3	EVS*WP → KH	0.050	0.027	2.039	0.045	Supported
H4	SEPR*WP → KH	0.079	0.030	2.659	0.008	Supported

The workplace friendship significantly moderates the slope for the relationship between EVC and Knowledge hiding. The slope is given in Figure 3.

**Figure 3:** A slope for ethical value congruences (EVC) and workplace friendship (WP).

The slope between SEPR and knowledge hiding is significantly moderated by the IC but negative in direction. The slope is given in Figure 4.

**Figure 4:** A slope for lack of shared ethical priorities (SEPR) and WP.

## Discussion

The core objective of this research was to examine the impact of ethical conflict having two dimension ethical value congruences and lack of shared ethical priorities on knowledge hiding and investigate the workplace conflict. Four hypotheses were generated based upon the our proposed model. Data were collected from the employees working in colleges and universities of China. The results indicate that ethical conflict significantly impacts knowledge hiding at team level, which is consistent with the finding of previous studies (Boz Semerci, 2019). H_1_ proposed that there is significant relationship between ethical value congruence and knowledge hiding. The results empirically substantiate that ethical value congruence has a positive relationship with knowledge hidings. Although the relationship between ethical value congruence and knowledge hiding is significant, it is contradictory to the previous studies (Thorne, 2010). However, all these studies were conducted at the individual level but in this study we are measuring the concept at team level so there are certain other factors which may promote the knowledge hiding behavior among employees working in the team.

The article "Ethical Conflict and Knowledge Hiding in Teams: Moderating Role of Workplace Friendship in Education Sector" was retracted in 2025. Reasons: unreliable results or conclusions; a conflict of interest; concerns about the peer review; concerns about the citations.

H_2_ proposed that there is a relationship between lack of shared ethical priorities and knowledge hiding at team. The results empirically substantiate that ethical value congruence has a positive relationship with knowledge. This result is in accordance with previous studies (Thorne, 2010). Which suggested that if organization’s priorities for ethical behavior are not consistent with those of the employee which leads to decrease employees commitment toward their team and organization and they feel alienate from their team and organization. Consequently, in exchange, they feel resultant to share their knowledge with other team and adopt knowledge hiding, which decreases the performance of the team and the organization.

H_3_ proposed the workplace friendship moderating role in the relationship of shared ethical priories and knowledge hiding. The results are consistent with Guohao et al. (2021), which posit that there is a certain complication which is created because of workplace friendship (Ingram and Zou, 2008) resultantly, these complications effect the decorum of the organizations as employees goals are differentiated from their organizational goal. H_4_ anticipated moderating role of Workplace friendship in the relationship of Lack of shared ethical priorities and knowledge hiding. The results demonstrate that if workplace friendship exists in the organization, the relationship between shared ethical priorities and knowledge hiding gets weaker. These results validate with the finding of Yu et al. (2021).

### Theoretical and Managerial Implications

This study contributes in the body of literature in very important ways. It explores the two important dimensions of ethical conflict, that is, ethical value congruence and lack of shared ethical priorities. Similarly, Literature of knowledge hiding depicts that most of the studies examined the knowledge hiding behavior at individual level (Zhang and Min, 2021). Recent studies emphasized the need of knowledge hiding behaviors at the team level (Zhang and Min, 2021). We addressed the research gap and explore the knowledge hiding behavior at the team level. Prior studies indicate that there is no study examine the impact of ethical conflict and knowledge hiding. Thus this study found that there is a significant impact of ethical conflict on knowledge hiding behavior of employees. Similarly, this study uses the theoretical lens of social exchange theory and absorptive capacity to examine the impact of ethical conflict on knowledge hiding. Furthermore, this result indicates that workplace friendship moderates the relationship between ethical conflict and knowledge hiding.

The article "Ethical Conflict and Knowledge Hiding in Teams: Moderating Role of Workplace Friendship in Education Sector" was retracted in 2025. Reasons: unreliable results or conclusions; a conflict of interest; concerns about the peer review; concerns about the citations.

This research study provides several significant practical implications for policymakers, practitioners and education experts. This study highlighted that ethical conflict leads to adverse outcomes, such as promoting the knowledge hiding behaviors. Thus, the organization’s top management should devise and comprehensive policies to align the organizational value with the employees’ values. The organization should focus on training and development of their staff. Comprehensive training and orientation sessions should be conducted to teach the organization culture and values among the employees. Management should make their efforts to make organizational culture flexible and employees friendly. The critical action should be taken to mitigate the knowledge hiding behavior among the staff. This is possible only through awareness and rewards package. Special incentive program should be designed to promote knowledge sharing behavior in the staff.

Hence, organization management and leadership should ensure TQM practices in workplace. Along with this, knowledge sharing and internal service quality also significant importance to improve the project performance. Thus, organizational leadership also focus on these two aspects. Extensive training programs and seminars should be commenced to build the knowledge share behaviors among the staff. Incentive programs should be designed in considering of these aspects. Similarly, this study implies the significant moderating role of workplace friendship thus education organization and top management should focus on encouraging workplace friendship behavior in the education industry.

### Limitations

Although this study has made several contributions but this study is not without limitation which should be address in the future studies. Firstly, the current study collect data from single sources which might be risk of common method biasness thus future studies should collect data from multiple sources to reduce the chances of common method biasness. Secondly, sample size of this study is not sufficient to generalize result therefore future studies should collected data from large population so the result should generalize over whole population. Lastly, this research is cross-sectional in nature due to shortage of time and limited resources. The sampling technique used for obtaining data collected was convenience sampling because it was not pragmatic to collect data through formal ways. Further studies should utilize most rigorous sampling technique to get better result. Along with this, future studies should add more mediators and moderator between ethical conflict and knowledge hiding.

The article "Ethical Conflict and Knowledge Hiding in Teams: Moderating Role of Workplace Friendship in Education Sector" was retracted in 2025. Reasons: unreliable results or conclusions; a conflict of interest; concerns about the peer review; concerns about the citations.

## Conclusion

Drawing on social exchange theory and affective event theory, this study examines the impact of two dimensions of ethical conflict, that is, shared ethical priorities and ethical value congruence, on knowledge hiding behavior at team level and investigates the moderating role of workplace friendship between this relationship. This study implies that if the ethical values of individual are contradictory to the organization’s value then conflict arises. Resultantly, individual feel reluctant to share their knowledge with their colleagues. Similarly, if the workplace friendship culture prevails in the organization then it is possible to mitigate the knowledge hiding behavior at team level. Data were collected from the 450 employees working in the colleges and universities of China. PLS-SEM technique was adopted to measure the theoretical framework of this study. The finding of this study indicates that there is a significant impact of ethical conflict on knowledge hiding. Similarly, workplace friendship moderates this relationship.

## Data Availability Statement

The original contributions presented in the study are included in the article/supplementary material, and further inquiries can be directed to the corresponding author.

## Ethics Statement

The studies involving human participants were reviewed and approved by Hunan University of Science and Technology (HUST), China. The patients/participants provided their written informed consent to participate in this study. The study was conducted in accordance with the Declaration of Helsinki.

## Author Contributions

SX: conceived, designed the concept, collected and wrote the paper. The author read and agreed to the published version of the manuscript.

## Conflict of Interest

The author declares that the research was conducted in the absence of any commercial or financial relationships that could be construed as a potential conflict of interest.

## Publisher’s Note

All claims expressed in this article are solely those of the authors and do not necessarily represent those of their affiliated organizations, or those of the publisher, the editors and the reviewers. Any product that may be evaluated in this article, or claim that may be made by its manufacturer, is not guaranteed or endorsed by the publisher.
